RETRACTED

# Peripheral Cytokines as a Chemical Mediator for Postconcussion Like Sickness Behaviour in Trauma and Perioperative Patients: Literature Review

**DOI:** 10.1155/2014/671781

**Published:** 2014-04-28

**Authors:** Yasir Rehman, Nadia Rehman, Riaz Rehman

**Affiliations:** ^1^Neuro Science, Division of Neurology, Department of Medicine, Mc Master University, Hamilton, ON, Canada; ^2^CCRA, Mc Master University, Hamilton, ON, Canada; ^3^Gomal University, D I Khan, Pakistan; ^4^Windsor University, St Kits, Anguilla

## Abstract

Besides brain injury and systemic infection, cognitive and concussion like sickness behaviour is associated with muscular trauma and perioperative patients, which represents a major obstacle to daily activities and rehabilitation. The neuroinflammatory response triggers glial activation and consequently the release of proinflammatory cytokines within the hippocampus. We review clinical studies that have investigated neurocognitive and psychosomatic symptoms related to muscular trauma and in perioperative conditions. These include impaired attention and executive and general cognitive functioning. The purpose of this literature review is to focus on the systemic inflammation and the role of proinflammatory cytokines IL1, IL6,and TNF and other inflammatory mediators which mediates the cognitive impairment and induces sickness behaviour. Moreover, this review will also help to determine if some patients could have long-term cognitive changes associated with musculoskeletal injuries or as a consequence of surgery and thereby will lead to efforts in reducing that risk.

## 1. Introduction

Neurocognitive and concussion like sickness behaviour is a cluster of signs and symptoms following a traumatic brain injury or systemic infections [1]. These signs and symptoms such as headaches, dizziness, neuropsychiatric manifestations, and cognitive impairment are usually deficits in somatic and behavioural domains [2]. Literature shows that impairment in mental functions following traumatic event has a common biological origin in the form of neuroinflammation [3], which triggers a complex cascade of events such as activation of inflammatory cells and proteins and expression of cytokines [1, 3]. These inflammatory events lead to unavoidable brain damage such as alteration in hippocampal cholinergic function, which mediate changes in cognition and behaviour [1]. The circumstantial data suggests that proinflammatory cytokines may play a role in instigating long-term cognitive and depressive like behaviour by infiltrating neurological tissue in individuals [4, 5].

Cytokines have been studied to assess neurologic injury in various surgeries, traumas, infections, strokes, neuropsychiatric disorders, and autoimmune diseases such as multiple sclerosis [6, 7]. Postoperative cognitive deficits such as impairment of recent memory, concentration, language comprehension, and social integration have been reported in 25.8% of patients one week after the surgery and in 9.9% of patients three months after the surgery [8]. Newman et al. in 2001 [9, 10] reported that neurocognitive decline (NCD) is a common complication with a prevalence up to 50%. The postoperative cognitive deficits also depend on type of surgery, medications, and preexisting medical conditions. The cognitive deficits after trauma and after operation are associated with significant decline in patient's quality of life, prolonged hospitalization, and increased overall morbidity and mortality [7].

RETRACTED

In our opinion the overexpression of proinflammatory cytokines in muscular trauma directly influences the hippocampal dependent long-term potentiation and memory, that is, spatial memory, attention, executive function, object recognition, and contextual fear conditioning and synaptic plasticity. The higher cognitive processes rely heavily on learning and memory processes but their relationship with cytokines remains poorly understood.In this review we proposed cytokines and neuroinflammatory model of neurocognitive symptoms in trauma situation. The main research question of the current study is whether there is an association of muscular IL-6, IL-1, TNF, and other inflammatory mediators with neurocognitive impairment when released as result of the trauma or perioperatively. Our main hypothesis is that IL-6, TNF, IL-1, and other inflammatory mediators released in muscular, orthopedic trauma or perioperative conditions are associated with neurocognitive impairment and concussion like illness and are not merely the result of anesthesia or medications. The purpose of this review is to systematically evaluate the literature and to clarify this entrenched belief. In our opinion, this hypothesis has implications for the pathogenesis and treatment of cognitive psychosomatic deficits in the trauma and postoperatively.

## 2. Evidence Acquisition and Synthesis

The Mc Master University database using Ovid/MEDLINE database was searched for articles published between 1946 and July 2013 using the following combination of the terms: cognitive impairment, traumatic brain injury, cytokines (IL-1, IL-6, IL-8, and TNF-a), neuroinflammation, concussion like symptoms, blood brain barrier, systemic inflammatory response, and polytrauma. All articles were published in peer-reviewed journals, reporting original data on cytokines and systemic inflammatory response. All the key words were used by using mesh words and were initially combined by using “OR.” The words in each category such as neuroinflammation, cytokines, and cognition were then combined using “AND.” Our initial data search showed gave us 303447 in neurocognitive domains, 396588 in muscle and peripheral injury group, and 715522 in neuroinflammation category. On combing with “AND” the initial result was limited to 224 published articles. The selection was further limited to human and English language, which gave us 172 published articles. For articles review, I followed the PRISMA and “second chapter of 3rd edition of clinical epidemiology in clinical research.” We excluded all the review articles and animal study models. We also excluded articles that studied cytokines response in nontraumatic causes such as stroke, SAH, HIV, or infections, cancers, and immunotherapy. Out of those 172 published articles, 9 articles were selected to support the systemic effects of the cytokines, 23 articles to support the cognitive and behavioural symptoms that can be explained secondary to cytokines, and 21 articles to support the evidence that cytokines are related to peripheral trauma. 

RETRACTED

*Summary of the Important Literature*. Clinical studies of peripheral blood or autopsy specimens show elevated increases in cytokines TNF-*α*, IL-1*β*, and IL-6 in serum and cerebrospinal fluid (CSF) of patients with mild to moderate late-onset Alzheimer disease (AD) [11, 12]. Simultaneously, age-associated changes in glial reactivity may predispose individuals to exacerbated neuroinflammatory cytokine responses that are permissive to cognitive and behavioural complications [7].

Similar cognitive and behavioural symptoms are reported in perioperative process and trauma [7]. It has been suggested that surgical tissue trauma and stress response induce perioperative nonspecific inflammatory response. IL-6 response to injury is robust, being demonstrated across many types of injuries [13] including muscle, skin, bone, lung, and fat [14]. Elevated IL-6, in a lumbar decompression surgery, in the first 24 hours is associated with cognitive deficits and prolonged hospital stay [15]. Hogevold et al [16] reported that chemical mediators particularly Il-6, CK, TNF-alpha and IL-1 are strongly correlated with muscular injury response and surgery, which supports our opinion. Li et al. [17] found that only elevations in IL-6, S100b, were associated with cognitive impairment and delirium, following hip fracture surgery [17, 18]. Perioperative increase in CRP and inflammatory cytokines such as IL-1 and -10 is associated with neurocognitive deficits (NCD) in patients after cardiopulmonary bypass [6, 19]. Kálmán et al. [20] reported elevated levels of inflammatory biomarkers in CSF as predictor of cognitive decline in coronary artery bypass surgery.

RETRACTED

Haas [21] has found that professional amateur sports athletes, whiplash, and polytrauma patients show neurocognitive weakness in the absence of brain injuries, gram negative pathogenesis, infections, cerebrovascular disease, and neurodegeneration. Elevated serum IL-6 has been shown to correlate with multiorgan failure and death in polytrauma patients [22, 23]. Hensler et al. [24], Alexander [25], Gunstad and Suhr [26], and Iverson and Lange [27] reported increased serum concentrations of proinflammatory cytokines, including IL-6, in patients with multiple injuries and a high prevalence of the neurocognitive and behavioural symptoms (see Table 1).

In various diseases states, and behavioral syndromes, inflammatory biomarkers have been found to be positively correlated with fatigue [46–50, 61, 62], sleep disturbances and irritability [52–54, 63], and irritability [51]. Negative changes in mood and impaired learning and memory are significantly correlated with increases in IL-6, TNF-*α*, and IL-1 [17, 29].

On contrary to the above, there are studies that show that a decrease in peripheral systemic inflammation reduces the neuroinflammation, thus decreasing the sickness induction behaviour and improving cognitive functions. Acute and chronic exercises have anti-inflammatory effects, reducing levels of proinflammatory cytokines and CRP. Exercise as a therapy for PCS seems to be supported by the fact that young athletic individuals have evidence of anti-inflammatory mediators that oppose the actions of IL-6 and TNF-*α* [4]. Nonsteroidal anti-inflammatory drug (NSAIDs) user has a lower risk and progression of AD and NSAIDs are already being explored as a treatment for depression [64]. Acetylsalicylic acid has already been shown to accelerate remission in individuals who are not responsive to SSRIs [65]. Interestingly, a recent report from Tobinick and Gross shows a rapid cognitive improvement following perispinal etanercept (a potent TNF-*α* antagonist) administration in an Alzheimer patient [7].

## 3. Data from Preclinical or Animal Studies

Noninfectious systemic inflammatory markers have been independently associated with impaired cerebral blood flow [66]. Animal inflammatory models suggest focal dysregulation in cerebrovascular flow in areas important to memory, such as the hippocampus [67]. Animals treated with cytokines, such as IL-1*β* or TNF-*α* or IFN-1*β*, exhibit “sickness behaviours,” including reduced locomotor activity, diminished social interactions, and diminished consummatory behaviours [68]. Transgenic mice expressing IL-6 in glial cells show ataxia, seizures, and extensive neurodegeneration [69]. The animal model study shows differences in regional uptake such as the TNF uptake. TNF uptake into the hypothalamus is 9 times faster than into the parietal cortex and is not taken up by the striatum or the midbrain. Differences also exist between brain and spinal cord transport rates; for example, the transport rate of IL-1 into the spinal cord is about 80% of the brain. Variations also occurred among the regions of the spinal cord. The cervical spinal cord was the region with the fastest transport rate for both interferon (INF) and TNF [70]. Cauli et al. [71] reported that ibuprofen restored learning ability in rats with hepatic encephalopathy induced by portacaval shunts. The posttraumatic blood levels and pharmacological therapy aimed at enhancing the protective cytokines and inhibiting the damaging cytokines have shown improved survival rates in experimental animals [3].

RETRACTED

## 4. Discussion

### 4.1. Peripheral Trauma-Cytokine-Neurocognitive and Behavioural Model

Trauma initiates immune reaction, circulating T Cells activation, proliferation, and cytokines expression [72]. Once activated, cytokines exert inflammatory and compensatory anti-inflammatory process and wound repair and healing mechanisms [73–75]. However their dysregulation and prolonged and excessive inflammatory response to pathophysiological insults lead to secondary injury, immune alteration, and multiorgan failure [76]. Release of cytokines also depends on the extent of the injury or trauma. A person is more prone to develop cognitive decline following a major muscular injury or surgery as compared to minor injury or laparoscopic surgery [77, 78].

After the major trauma or surgery, immune cells such as CD+4 T lymphocytes, peripheral blood mononuclear cells (PMBC), and macrophages are activated [79, 80]. Cytokines are derived from type I and II CD+4 helper T cells (HT). Type 1 CD+4 HT promote cytokines IL-1-alpha and -beta, IL-2, IFN-*γ*, and TNF. Type II CD+4 (HT) secrete cytokines such as IL-4, IL-6, and IL-10 [81]. A balance between the CD+4 (I and II) cells is critical to maintain immune homeostasis; however, imbalance between the two cell lineages is responsible for antigen presentation to peripheral blood mononuclear cells (PMBC), increase in expression of TNF, IL-1, and IL6, and alteration in antigen presentation and mitogen in trauma patients [78, 82, 83]. These systemic cytokines are involved in cell-to-cell communication and are partially propagated by systemic immune response system (SIRS) and multiorgan dysfunction (MODS) [22].

The brain is an immunologically active organ and is in direct communication with the immune and endocrine systems [12]. Human brain has IL-1, IL-2, IL-6, and TNF-cytokine receptors at frontal cortex, hippocampus, hypothalamus, cerebellums, and cerebrovascular endothelium [12]. The hippocampal formation and the dentate hilar region are differentially sensitive to injury relative to other regions of the brain, even in the absence of hypoxia or elevated intracranial pressure or without actual neuronal cell death [1].

RETRACTED

Cytokines alert human brain through immunoneuropsychiatric (INP) cascade, secondary to peripheral inflammatory process due to injury [84]. In brain, the peripheral cytokines act as a second messenger and activate calcium, which triggers the blood brain barrier (BBB) damage and destruction of tight junctions [77, 85]. There are two mechanisms of cytokines transport across the blood brain barrier. First is direct or active transport of cytokines across the blood brain barrier through cytokines receptors. Second is indirect transport diffusion at the circumventricular region (CVO), where the BBB is incomplete [77]. CVO also prevents cytokines diffusing out. Another indirect mechanism of peripheral cytokines transport is via vagal nerve stimulation of nucleus tractus solitarius (NTS) in brain stem and then preoptic area of hypothalamus [12, 86, 87] (Figure 1).

Once in brain, the peripheral cytokines particularly IL-1 stimulate the microglia, which further stimulates the endogenous or central cytokines (IL-1, IL-6, and TNF-*α* production [77]). Once in the brain, both central and peripheral cytokines act through similar mechanism. Cytokines are pleotropic mediators and exert their effects through complex immune cascades, interaction with complement system, altered excitotoxic glutamate transmission, abnormal neurotransmission, oxidative stress, and nitric oxide production, leading to apoptotic neurodegeneration [88–90]. Neuroinflammation influences neuronal and axonal survival [91–95] and alters the central noradrenergic, dopaminergic, tryptophan, and serotonergic neurotransmission in the hypothalamus hippocampus [96]. The cell debris and central stress further induce the central expression of IL-1, IL-6, and TNF in a vicious cycle [97, 98]. Cytokine known as mediator of physical and psychological stress also alters the hypothalamic-pituitary-adrenal axis and cortisol regulation [99]. Peripheral cytokines also exert indirect effects on the cognitions such as disrupting sleep regulation, micronutrient deficiency by appetite suppression, and endocrine interactions [70].

On the other hand, cognitive and behavioural stresses also influence cytokine production and alter the immunologic equilibrium [100]. Thus central and peripheral cytokines mediated processes proceed in parallel to affect cognition. As a mediator of bidirectional communication between CNS and the peripheral immune system, systemic inflammatory reactions can influence brain function and conversely CNS processes may affect distant organs (Figures 2 and 3).

RETRACTED

The most important and well-studied cytokines after peripheral trauma are IL-6, tumour necrosis factor-alpha (TNF-*α*), IL-1*β*, IL-2, IL-8, and IL-4 and recently IL-18, IL-12, and IFN-*γ* [15, 30]. In the periphery, IL-1, IL-6, and TNF are typically considered proinflammatory, whereas IL-4, IL-10, and IL-13 are typically considered anti-inflammatory [12]. The proinflammatory cytokines particularly IL-6 are the acute-phase response proteins that contribute to the development and resolution of signs and symptoms of acute and chronic inflammation after soft tissue injury [93, 101]; see Table 2. 

*IL-1*. Peripheral IL-1 plays important role in neuroendocrine modulation, proliferation, and expression of microglia [3]. Peripheral IL-1 also alters central release and turnover of norepinephrine, serotonin, dopamine, and cholinergic neurotransmission [102]. IL-1 also affects hippocampal neurons and the synaptic plasticity [103–106], thus inhibiting the long-term potentiation (LTP) [107]. 

*IL-6.* Peripheral IL-6 is acute-phase protein, increases vascular permeability, and induces lymphocytic activation. IL-6 once in brain induces microglia and astrocyte activation, which further triggers the release of proinflammatory cytokines [108]. IL-6 alters the neuroendocrine neurotransmission, hypothalamic-pituitary-adrenal (HPA) axis, and ACTH release [109]. IL-6 alters the noradrenergic and serotonergic neurotransmission [109]. IL-6 impacts cognitive function via effects on synaptic plasticity [17, 110], decline in learning, memory, and long-term potentiation (LTP) [17].

*TNF-Alpha. *Tumor necrosis factor has neurodegenerative effects [111]. TNF has a direct effect on the LTP and synaptic plasticity [56]. It exerts its effects by activating caspases [112, 113], which activate the death signalling pathway [56] via glutamate excitation [56]. TNF alters the synaptic efficacy by upregulating surface expression of  *α*-amino-3-hydroxy-5-methyl-4-isoxazolepropionic (AMPA) receptors [114] and phosphatidylinositol 3 (PI3) kinase-dependent processes [115], thus causing a decrease in the synaptic inhibition and cognitive impairment [56]. 

*CRP.* CRP is the inflammatory marker and correlates with IL-6 secretion. CRP is associated with inflammation, impaired endothelial function, and cerebral amyloid deposits in areas important to memory, such as the hippocampus [116]. CRP is associated with memory, visuospatial impairment, and disruption of frontal subcortical pathways [117]. 

RETRACTED

*IL-2.* IL-2 alters dopaminergic transmission and impairs the spatial memory performance via hippocampal neurodegeneration and suppression of long-term potentiation [118]. Immunotherapy, using IL-2, induces a depressive like state that may be attenuated by antidepressant treatment [41].

*IFN-γ*. * IFN-gamma* is associated with more general cognitive dysfunction, confusion, psychomotor slowing, parasthesia, visual disorientation anxiety, and depression [119]. IFN induces IL-1, TNF secretion, and depletion of serotonin, which contributes to cognitive and behavioural effects [120].

As previously mentioned, brain regions particularly dorsolateral frontal cortex, hippocampus, hypothalamus, cerebellums, and cerebrovascular endothelium are susceptible to cytokines and neuroinflammation. These brain regions are involved in memory, learning, executive functions, and personality. Therefore neuroinflammation in these regions leads to neurocognitive and behavioural changes. The manifestations of sickness behaviour include increased somatic complaints, lethargy, sleep disruption, reduced social activity, reduced mobility, anhedonia, decreased learning, anorexia, decreased libido, and neuropsychiatric side effects including depressed mood, poor motivation, and impaired thought processing [70]; see Table 3. Almost all the signs and symptoms of disease, including altered behaviour and neuropsychiatric phenomena, can be accounted for by the actions of immune cell and peripheral cytokines secretions [93]. These profound discoveries have recently been applied to psychosocial disease, schizophrenia [35, 121], and depression [121, 122] yielding completely new models for the etiology of these unexplained diseases [123]. There is abundant evidence that peripheral inflammation can worsen or cause the axonal injury and exacerbate preexisting psychiatric disorders as well as the new onset of mood disorders (depression and mania), anxiety disorders, and psychotic disorders [1].

Overall, based on the above literature reviews, the peripheral inflammatory response interferes with cognitive function as evidenced by abnormal memory, learning, and inability to develop long-term potentiation in hippocampus [7]. Given that similar symptoms may be seen in such diverse situations as perioperatively, after orthopedic or general trauma, perhaps it is time to consider PCS as merely one of many states in which there is an elevation of inflammatory cytokines. This hypothesis certainly opens a room to develop or determine inflammatory markers that might be helpful to address the cognitive weakness in postoperative and trauma patients and to study potential prediction of postsurgical or posttrauma risks and complications.

RETRACTED

Currently, PCS or sickness behaviour such as neurocognitive and behavioural deficits is treated based on the specific symptoms primarily supportive to the individual [124] and as such not treating the underlying cause [11]. Despite ongoing research, little progress has been achieved in terms of prevention or management of this problem, largely because of an incomplete understanding of the pathophysiology of cognitive impairment, which is essential to improve outcomes. In our opinion, some aggressive anti-inflammatory measures (including inflammatory cytokines antagonists or NSAIDs) may improve cognitive function in cognitive deficient subjects, particularly in trauma and perioperative patient. In our opinion the same will also be true for the PCS patients and may prevent the long-term neurologic sequelae of TBI, systemic inflammation, including cognitive impairment.

## 5. Conclusion

On the basis of the above overview, we believe there is sufficient clinical and research evidence to suggest clearly that cognitive impairment is not only limited to concussion, systemic infections and neurodegeneration. Furthermore, most PCS symptoms can be explained with current evidence by increased levels of cytokines such as IL-1*β*, IL-6, TNF-*α*, and IFN-*γ*, which are all important cytokines after trauma. Peripheral cytokines as those due to muscular injury or orthopedic trauma can influence neurotransmission and cause cognitive deficits. There is abundant evidence that there are cytokine-mediated interactions between neurons and glial cells, subserving cognition (e.g., cholinergic and dopaminergic pathways), and can modulate neuronal and glial cell function to facilitate neuronal regeneration and contribute to cognitive impairment.

## Figures and Tables

**Figure 1:** Release and activation of peripheral cytokines from PMBC; mechanism of cytokines transport across the blood brain barrier; IL-1, IL-6, and TNF after crossing BBB stimulate microglia to secrete endogenous cytokines as well as affect neuronal cell/transmission directly. (PMBC—peripheral mononuclear blood cells, MODS—multiorgan dysfunction syndrome, TNF—tissue necrosis factor, IL-1—interleukin 1, and IL-6—interleukin 6).

**Figure 2:** Vagal nerve stimulation and effect on hypothalamus-pituitary-adrenal axis; peripheral cytokines after crossing the blood brain barrier (BBB) also directly affect hypothalamus-pituitary-adrenal axis.

**Figure 3:** Two-way communication of peripheral and central cytokines (peripheral cytokines affect central cytokines, whereas central stress behaviour affects the peripheral cytokines release).

RETRACTED

**Table 1:** The literature overview that studied cytokines release in condition other than TBI, infections, cardiac conditions, HIV, strokes, cerebrovascular conditions, cancers, immunotherapy, MS, or any condition in which the neurocognitive dysfunction is expected.

Reference	Systemic condition	Cytokines/inflammatory markers	PCS symptoms
Lenz et al. 2007 [22]	Polytrauma,	IL-6	Cognitive impairment
Hergenroeder et al. 2010 [23]	Orthopedic trauma, polytrauma	IL-6	Cognitive impairment
Hensler et al. 2002 [24]	Polytrauma	IL-6	Systemic inflammatory response syndrome
Li et al. 2012 [17]	Fracture surgery, postoperative hip replacement	IL-6, S-100 B	Cognitive impairment and delirium
van Munster et al. 2010 [18]	Fracture surgery	IL-6, S-100 B	Cognitive impairment and delirium
Dowlati et al. 2010 [28]	Meta-analysis, polytrauma	TNF-*α* and IL-6	Depression
Wright et al. 2005 [29]	Polytrauma	IL-6, TNF-*α*,and IL-1	Changes in mood, impaired learning and memory
Wilson et al. 2002 [12]	Physical stress	IL-6	Physical or psychological stress
	Autopsy specimen	IL-1, IL-6, or TNF-a	Mild to moderate late-onset AD
Bastian et al. 2008 [30]	Trauma	IL-1*β*, IL-6, TNF-*α*, and IFN-*γ*	Systemic inflammatory response syndrome
Harrison et al. 2009 [138]	Trauma	IL-6, IL-1, and TNF	Changes in mood, impaired learning and memory
Haas 1996 [21]	Professional amateur sports athletes	IL-6, IL-1, TNF	PCS like symptoms and long-term depressive like behaviour
Kumbhare et al. 2009 [15]	Lumbar decompression surgery	IL-6	Cognitive impairment, systemic inflammatory response syndrome
Haensel et al. 2009 [31]	Obstructive sleep apnea	IL-6, TNF, TNF-R1	Cognitive functioning, mood, and sleep
Heffner et al. 2012 [32]	Acute stress	IL-6	Cognitive tests, sleep quality, depressive symptoms, perceived stress, and loneliness
Tsaoussoglou et al. 2010 [33]	Excessive daytime sleepiness, inflammation, and metabolic abnormalities.	(IL-6, TNF-alpha, CRP)	Sleep disruption, fatigability
van de Vyver and Myburgh 2012 [34]	Biopsy	IL-1, IL-6, IL-10, CK, TNF, LDH,	Systemic inflammatory response syndrome, cognitive impairment
Smith 2000 [35]	Overtraining syndrome (OTS)	IL-1-beta and/or IL-6 and/or TNF-alpha	Systemic inflammatory response syndrome
Perl et al. 2003 [14]	Blunt trauma	IL-6, IL-8	Systemic inflammatory response syndrome
Flohé et al. 2007 [36]	Soft tissue trauma, hip surgery	Heat shock protein, TNF-alpha	Systemic inflammatory response syndrome
Barr et al. 2004 [37]	Work-related musculoskeletal disorders	IL-1, CTGF	Decreased locomotor function
Strecker et al. 2003 [38]	Blunt chest trauma	IL-8, IL-6, and CK	Systemic inflammatory response syndrome

RETRACTED

**Table 2:** The overview of common but important inflammatory markers involved in systemic inflammatory response and neurocognitive compromise.

Inflammatory marker or cytokines (peripheral)	Reference	Associated conditions	Common symptom associated	Mechanism	Effect on other cytokines (if +)
IL-6	Hergenroeder et al. 2010 [23]	Orthopedic, muscular injury, and surgery	Depression, memory impairment	HPA axis, alters NE, serotonin, dopamine, and cholinergic neurotransmission	Production of other cytokines and propagation of the inflammatory response

TNF-*α*	Melanie Lancette-Hebert et al. 2007 [139] Lenz et al. 2007 [22]	Surgery, muscle injury, and depression,	LTP and synaptic scaling	Generation of free radicals such as NO, chronic hyperexcitability, and alterations in gene expression	Production of other cytokines and propagation of the inflammatory response

IL-1*β*	Namas et al. 2009 [3]	Muscular injury, surgery	Inhibits the long term potentiation (LTP), synaptic plasticity	Proliferation of microglia, alteration of NE, serotonin, dopamine, and cholinergic neurotransmission	Synergistic action with other proinflammatory cytokines such as TNF-*α*

CRP	Xie et al. 2009 [7]	Postoperative, muscular, and orthopedic injury, cardiac surgery	Memory and visuospatial impairment	Endothelial function, disruption of frontal subcortical pathways	IL-1, IL-6, TNF-a, IL-B, IL-10, and serum Tau protein

S-100 B	Hayakata et al. 2004 [39] Sedaghat and Notopoulos 2008 [40]	Muscular injury	Cognitive dysfunction	Neurotoxic at higher concentration	IL-6, IL- 8, IL- 10, IL-1, and TNF-*α*

IL-2	Anisman et al. 2002 [41]	Depressive state	Impaired spatial memory performance	Dopaminergic transmission, hippocampal LTP	

INF	Anisman et al. 2002 [41]	Depressive state	Cognitive dysfunction, confusion, and psychomotor slowing	Depletion of serotonin	IL-1, TNF

**Table 3:** The PCS symptoms explained based on the cytokines.

PCS symptoms	Systemic illness	Reference	Cytokines associated
Headache	Migraine headaches	Munno et al. 2001 [42]	IL-10
	Review articles	Martelletti 2000 [43]	IL-1B, TNF-a
		Williamson and Hargreaves 2001 [44]	CGRP, calcitonin, and TNF-a

Fatigue	CARDIA	Cho et al. 2009 [45]	CRP
	WBC	Raison et al. 2009 [46]	CRP
	Cancer patients	Schubert et al. 2007 [47]	CRP, IL-1, and IL-6
	Coronary heart disease	Janszky et al. 2005 [48]	CRP, IL-1, and IL-6
	Rheumatoid arthritis	Davis et al. 2008 [49]	CRP, IL-1, and IL-6
	Multiple sclerosis	Heesen et al. 2006 [50]	IFN-*γ*, TNF-*α*

Irritability	Verbal aggression and irritability	Ahren-Moonga et al. 2008 [51]	IL-6

Insomnia or sleep disturbance	Excessive daytime sleepiness, sleep apnea, narcolepsy, and idiopathic hypersomnia	Vgontzas and chrousos 2002 [52]	IL-6 and/or TNF-a
	Sleep deprivation	Vgontzas and chrousos 2002 [52]	IL-6, cortisol
	Hemodialysis	Erten et al. 2005 [53], Chiu et al. 2009 [54]	IL-B,

Reduced tolerance to stress, emotional excitement	General stressors	Anisman et al. 2002 [41]	IL-1*β*, TNF-*α*
	Mood	Brydon et al. 2009 [55]; Himmerich et al. 2006 [11]	IL-6, IL-1, and TNF-a

Cognitive and memory difficulties	Hippocampal dependent memory	McAfoose and Baune 2009 [56]	IL-1*β*, TNF-*α*
	Cognitive functions	McAfoose and Baune 2009 [56]	IFN-*γ* (cognitive dysfuntion), IL-6 (impaired learning and memory), and IL-2 (spatial working memory)

Anxiety, depression, personality changes, and apathy	ACS	Joska and Stein 2008 [57], Poole et al. 2011 [19]	
	Immunotherapy	Anisman et al. 2002 [41]	IL-2, IFN-1B
	Systemic trauma, depression	Wright et al. 2005 [29], Reichenberg et al. 2001 [58], and Dowlati et al. 2010 [28]	IL-6
	Systemic trauma	Meares et al. 2008 [4]	IL-6, TNF-a

Dizziness	Headaches, migraines	Humphriss and Hall 2011 [59]; Calhoun et al. 2011 [60]	IL-1B, TNF-a, and IL-10
